# A first-in-human study investigating biodistribution, safety and recommended dose of a new radiolabeled MAb targeting *FZD10* in metastatic synovial sarcoma patients

**DOI:** 10.1186/s12885-018-4544-x

**Published:** 2018-06-08

**Authors:** Anne-Laure Giraudet, Philippe Alexandre Cassier, Chicaco Iwao-Fukukawa, Gwenaelle Garin, Jean-Noël Badel, David Kryza, Sylvie Chabaud, Laurence Gilles-Afchain, Gilles Clapisson, Claude Desuzinges, David Sarrut, Adrien Halty, Antoine Italiano, Masaharu Mori, Takuya Tsunoda, Toyomasa Katagiri, Yusuke Nakamura, Laurent Alberti, Claire Cropet, Simon Baconnier, Sandrine Berge-Montamat, David Pérol, Jean-Yves Blay

**Affiliations:** 1 Department of Nuclear Medicine, LUMEN, Centre Léon Bérard, 28 Rue Laennec, 69008 Lyon, France; 2 Medical Oncology Department, Centre Léon Bérard, Lyon, France; 3 OncoTherapy Science, Kawasaki City, Kanagawa Prefecture Japan; 4 Clinical Research Platform, DRCI, Centre Léon Bérard, Lyon, France; 5 Université Lyon 1, CNRS, LAGEP UMR 5007, HCL, Lyon, France; 6 Pharmacy, Centre Léon Bérard, Lyon, France; 7 Biological sample Management Platform (PGEB), Centre Léon Bérard, Lyon, France; 8 INSA-Lyon, Université Lyon 1, CNRS, Inserm, CREATIS UMR 5220, U1206, Lyon, France; 9 Institut Bergonié, Bordeaux, France; 10 Division of Genome Medicine, Institute for Genome Research, The University of Tokushima, Tokushima, Japan; 11 Laboratory of Molecular Medicine, Human Genome Center, Institute of Medical Science, The University of Tokyo, Tokyo, Japan; 12 Present Address: Department of Medicine and Surgery, The University of Chicago, Tokyo, Japan; 13 Fédération de Recherche Santé Lyon-Est, CNRS UMS3453/INSERM US7, Lyon, France

**Keywords:** Synovial sarcoma, Radioimmunotherapy, Theranostic, First-in-human trial

## Abstract

**Background:**

Synovial Sarcomas (SS) are rare tumors occurring predominantly in adolescent and young adults with a dismal prognosis in advanced phases. We report a first-in-human phase I of monoclonal antibody (OTSA-101) targeting *FZD10*, overexpressed in most SS but not present in normal tissues, labelled with radioisotopes and used as a molecular vehicle to specifically deliver radiation to *FZD10* expressing SS lesions.

**Methods:**

Patients with progressive advanced SS were included. In the first step of this trial, OTSA-101 in vivo bio-distribution and lesions uptake were evaluated by repeated whole body planar and SPECT-CT scintigraphies from H1 till H144 after IV injection of 187 MBq of ^111^In-OTSA-101. A 2D dosimetry study also evaluated the liver absorbed dose when using ^90^Y-OTSA-101. In the second step, those patients with significant tumor uptake were randomized between 370 MBq (Arm A) and 1110 MBq (Arm B) of ^90^Y-OTSA-101 for radionuclide therapy.

**Results:**

From January 2012 to June 2015, 20 pts. (median age 43 years [21–67]) with advanced SS were enrolled. Even though ^111^In-OTSA-101 liver uptake appeared to be intense, estimated absorbed liver dose was less than 20 Gy for each patient. Tracer intensity was greater than mediastinum in 10 patients consistent with sufficient tumor uptake to proceed to treatment with ^90^Y-OTSA-101: 8 were randomized (Arm A: 3 patients and Arm B: 5 patients) and 2 were not randomized due to worsening PS. The most common Grade ≥ 3 AEs were reversible hematological disorders, which were more frequent in Arm B. No objective response was observed. Best response was stable disease in 3/8 patients lasting up to 21 weeks for 1 patient.

**Conclusions:**

Radioimmunotherapy targeting *FZD10* is feasible in SS patients as all patients presented at least one lesion with ^111^In-OTSA-101 uptake. Tumor uptake was heterogeneous but sufficient to select 50% of pts. for ^90^Y-OTSA-101 treatment. The recommended activity for further clinical investigations is 1110 MBq of ^90^Y-OTSA-101. However, because of hematological toxicity, less energetic particle emitter radioisopotes such as Lutetium 177 may be a better option to wider the therapeutic index.

**Trial registration:**

The study was registered on the NCT01469975 website with a registration code NCT01469975 on November the third, 2011.

## Background

Synovial Sarcomas (SS) account for 2.5–5% of all soft tissue sarcoma and affect all ages, but is most prevalent among adolescents and young adults (15–40 years of age) [1]. Therapy for patients with localized disease is based on surgery followed by external radiotherapy. Five-year overall survival rates range from 36 to 76%. Recurrences may be local (30–50%) or distant (40%), with lung being the most common site of distant metastases. Survival is better in children, possibly because of major biological differences between SS of adults and children [2]. In the setting of advanced disease, systemic chemotherapy with doxorubicin and/or ifosfamide is the standard of care. However, median overall survival becomes close to 12–18 months [3, 4]. Most targeted agents have failed to show significant activity except the *VEGFR* inhibitors [5], pazopanib [6], and more recently regorafenib [7]. Thus, therapeutic options in advanced SS remain an unmet clinical need.

In a study by Nagayama et al., 26 genes were found to be commonly upregulated in SS based on the genome-wide gene expression profiles of 13 SS cases by cDNA microarray, including Frizzled homologue 10 (*FZD10*) [8]. *FZD10* belongs to the Frizzled family of seven-pass transmembrane receptors for molecules in the Wnt signaling pathway. It was found to be overexpressed in SS samples and was almost absent in remaining normal adult tissues except the placenta [9]. Based on these findings, a specific monoclonal-antibody that targets the N-terminal extracellular domain of *FZD10* (MAb 92–13) was developed as a first step toward the development of an antibody-based therapy for SS [10]. In vitro, MAb 92–13 has only a weak antagonistic activity on cell growth and no/little antibody­dependent cell­mediated cytotoxicity and complement-dependent cytotoxicity. In vivo, when radiolabelled with Indium-111 (^111^In), it bound and accumulated in up to 5 days after IV injection in SS tumor cells overexpressing FZD10 (SYO-1) implanted in nude mice and not in FZD10 negative SS tumor cells (LoVo). This provided evidence for a specific binding. MAb 92–13 was proved to get internalized into tumor cells by confocal microscopy and flow cytometric (FACS) analyses. When it was radiolabeled with Yttrium-90 (^90^Y), a highly energetic beta emitter radioisotope, tumor shrinkage was observed in immunocompromised Balb-c mice bearing established FZD10-positive SS tumor subcutaneous xenografts (SYO-1 cell line), without significant toxicity [10]. Indeed, tumor volumes were markedly reduced immediately after treatment after a single administration of 3,7 MBq. Median time to tumor progression was 58 days in treated mice and 9 days in the control group.

All together, these preclinical data support the clinical development of an antibody targeting FZD10 as a specific tool for radionuclide delivery to synovial sarcoma cells. OTS has developed a radioimmunoconjugate humanized anti-*FZD10* Ab (OTSA-101) demonstrating high in vitro affinity for FZD10.

In the present report, we describe the results of a FIH, first in class phase I study evaluating the use of ^111^In-OTSA-101 and ^90^Y-OTSA-101 in patients with advanced synovial sarcoma following a theranostic approach.

## Methods

### Study population

Patients were required to have metastatic, histologically confirmed, synovial sarcoma, resistant to standard treatment, not amenable to therapy with curative intent (surgery or radiotherapy) and previously treated with doxorubicin and ifosfamide. Other key inclusion criteria were: measurable disease as per Response Evaluation Criteria in Solid Tumors version 1.1 (RECIST v1.1); Eastern Cooperative Oncology Group Performance Status (ECOG PS) ≤ 2, life expectancy ≥3 months, adequate organ function, left ventricular ejection fraction > 50%; normal pulmonary function with Force Vital Capacity (FVC) at least 60% and diffusing capacity or transfer factor of the lung for carbon monoxide (DLCO) of at least 50%, no positive human anti-mouse antibody (HAMA) or human anti-chimeric antibody (HACA) response.

### Study drug

Oncology Therapy Science (OTS) provided a humanized chimeric anti-FZD10 antibody (named OTSA-101) covalently bound to the chelating agent p-SCN-Bn-CHX-A”-DTPA at molecular ratio varying between 2.0 and 3.6 (i.e. number of DTPA molecules to one molecule of antibody). The thiocyanate (SCN) group of the linker reacts with the amino group of lysine of OTSA-101 and is able to chelate radionuclides with five carboxyl groups.

OTSA-101-DTPA was radiolabeled with Indium 111 (^111^In-OTSA-101- Step 1 Imaging part) or Yttrium 90 (^90^Y-OTSA-101- Step 2 Therapeutic Part). 275 MBq of high purity ^111^In-chloride (specific activity >185GBq/g indium) in diluted hydrochloric acid (Covidien, Petten, The Netherlands) or 370 MBq or 1665 MBq of 90Ychloride (IBA-Cis bio, Saclay, France) were added to 1.5 mg of OTSA-101-DTPA in the presence of sodium acetate buffer (0.2 M, pH 5) and was incubated 90 min at 37 °C. At the end of the labeling, 0.8 mg of EDTA-2Na were added in the mixture solution. The radiochemical purity (RCP) was assayed with a gamma isotope TLC analyzer (Raytest, Courbevoie, France) using ITLC-SG (Biodex Tec-control black, Biodex, NY, USA) and 0.9% sodium chloride solution as mobile phase. ^111^In-OTSA-101 or ^90^Y-OTSA-101 remained at the origin whereas unbound ^111^In migrated with an Rf of 0.9–1. The radiochemical purity (RCP) of radiolabeled OTSA-101-DTPA was required to be over 90% before injection.

OTSA-101 radiolabeled antibody was injected over a 30 min intravenous injection with follow-up of vital signs (blood pressure, pulse rate and temperature) every 15 min until the end of infusion, and 1, 2, 3, 5 and 8 h post-dose.

### Study design

This trial was an open-label, single center FIH, in Class Phase I study. The main aims were to evaluate the in vivo tumor binding ^111^In-OTSA-101 and the feasibility of a theranostic approach.

The design of the study was based on a theranostic approach. Indeed, this trial was divided in 2 steps: i) *During the first step, called imaging part*, patients received a single IV injection of ^111^In-OTSA-101- and the in vivo biodistribution of ^111^In-OTSA-101 was assessed using planar whole body and thorax-abdomen-pelvis hybrid Single Photon Emission Computed Tomography/Computed Tomography (SPECT-CT) acquisitions (Tandem Discovery NM/CT 670 from GE Medical Systems Ge DISCOVERY NM/CT 670) performed at 1, 5, 24, 48, 72, 144 h post-injection. Indium 111 is a Gamma emitter with a long physical half-life (67.4 h) allowing for repeated scintigraphies over few days to better assess OTSA-101 lesions radiotracer kinetic. ^111^In-OTSA-101 tumor uptake compared to normal tissues uptake were first assessed with a visual analysis using a 5 grades visual scale applied on SPECT-CT images: grade 0, no uptake; grade 1: less than background (mostly mediastinum); grade 2: equal to background; grade 3: greater than background but less than liver; grade 4: equal or greater than liver. A Steering Committee evaluated on a case by case basis for each patient if he/she can proceed to the therapeutic part based on tumor uptake grade: patients were deemed eligible for the 2nd step only if they had at least one tumor lesion demonstrating tracer uptake greater than mediastinum (i.e. Grade > 2, Fig. 1) and 2D estimated liver dose less than 20 Gy [11]. Indeed, liver demonstrated the highest tracer uptake as usually observed in radioimmunotherapy. In addition, patients displaying abnormal/unexpected biodistribution of ^111^In-OTSA-101, or demonstrating with safety concerns including abnormal bronchoscopy and/or clinical deterioration due to rapid disease progression were withdrawn from the study for other therapeutic plan; ii) *During the 2nd step, called therapeutic part*, 12 patients were to be randomized between two initial dose levels of ^90^Y: Arm A: 370 MBq versus Arm B: 1110 MBq. Then, based on safety and preliminary efficacy data, a third dose level was planned in 6 additional patients to be treated with 2220 MBq of ^90^Y-OTSA-101 (Arm C). The initial interval between the 2 parts of the trial was 28 days, but was reduced to 14 days considering the almost complete clearance (less than 50 ng/mL) of the antibody from the blood by day 14 after the infusion of ^111^In-OTSA-101. Of note, during the course of the study a protocol amendment was made to close the Arm A due to no clinical benefit observed in the first 3 patients and Arm C was never opened.

**Fig. 1:** Consort diagram

Finally, patients who achieved at least stable disease following 12 weeks of treatment were allowed to receive additional doses of ^90^Y-OTSA-101 (according to the randomisation arm) with a maximum of 4 doses per year.

### Clinical assessments

The clinical assessments included complete medical history, physical examination, ECOG PS, triplicate 12-lead ECGs, tumor imaging and standard laboratory assessments. Additional investigation included respiratory function tests (including CO diffusion assessment) and cardiac assessments. A bronchoscopy was added to the screening due to occurrence of hemoptysis and following the recommendations of iDMC. Toxicity was evaluated on clinical examination and laboratory assessments performed 1, 2, 4, 6, 12 weeks after the injection and every 3 months thereafter. All AE were graded according to the National Cancer Institute-Common Terminology Criteria (NCI-CTCAE) Tumor assessments were done at baseline, at weeks 6 and 12 and every 3 months thereafter. Tumor response was evaluated as per RECIST v1.1.

### Pharmacokinetic sampling (PK)

In the first step, blood sample collection for PK analysis was performed at 1, 5, 24, 48, 72, 144 h post-dosing with additional sampling at 7 days after the injection. In the 2nd step, PK sampling for OTSA-101 was performed 1, 5, 24, 48 h after the injection with additional sampling at 14 and 28 days after the infusion and during the end of study visit. In addition, blood sample collection for ADA was done for all patients at pre-dose and 7 days after injection during the first step and at pre-dose and 14, 28 days after the injection in the second step. All PK and ADA samples were analyzed by Altanbio (Nantes, France). The analytical method consists of Ligand Binding Assay (LBA) that used biotinylated anti-idiotypic OTSA-101 for capture and the same anti-idiotypic antibody conjugated to sulfo-TAG for detection. The SoftmaxPro v5.4 Molecular device software was used for regression, calculation of concentration and the Watson LIMS 7.2 software for pharmacokinetic calculation.

### Statistics

The sample size was set to screen patients for major toxicity occurring in a large portion of the target population. Especially, based on binomial probabilities, in 6 patients treated with a specific dose of ^90^Y-OTSA-101 there was a 90% probability of observing one or more patients with a toxicity event, if that event occurs in at least 32% of the target population. Cohorts of 6 patients were to be initially randomized to the first 2 doses of ^90^Y-OTSA-101 (370 or 1110 MBq of ^90^Y). Then, a 3rd dose level of ^90^Y was planned to be investigated. The total number of treated patients was expected to be 18, depending of the number of Limiting Event (Imaging Part) and the number of Severe Toxicity (Therapeutic) occurring.

The primary endpoint for imaging part (part 1) was the rate of Limiting Event defined as unacceptable/unexpected biodistribution of OTSA-101 and/or absence of tumor uptake. Secondary endpoints were to describe the PK and safety profile of ^111^In-OTSA-101. The primary endpoint for Part 2 was the rate of severe toxicities defined any of the following AE assessed as related to the study drug and graded according to National Cancer Institute Common Terminology Criteria for Adverse Events (NCI CTCAE) v4.0 criteria: i) Grade 4 hematological toxicity lasting more than 7 days; ii) Grade 3 hematological toxicity lasting more than 2 weeks; iii) Any clinical (i.e. non-laboratory related toxicity) non-hematological Grade 3, iv) Any persistent Grade 2 toxicity on end organs (liver, kidneys, lung, heart…). The secondary endpoints were the rate of objective response as per RECIST v1.1, the clinical benefit rate and duration of response as well as PK parameters.

The safety population consists of all patients who received OTSA-101 and the intent-to-treat population consists of all included patients. Due to the nature and design of the study, the statistical analysis had mainly descriptive. Categorical data were described using contingency tables with frequencies and percentages. The missing data were not taken into account in percentages. Quantitative data were presented using number of observations, mean, standard deviation, median, maximum and minimum values. The statistical software SAS® release 9.4 was used for the analyses.

## Results

### Patient characteristics and consort diagram

From January 2012 to June 2015, 20 patients with advanced/recurrent synovial sarcoma were enrolled in the Imaging part (See Fig. 1 and Table 1). Among them, 10 had insufficient tumor uptake making them ineligible for Part 2 and 10 patients have shown significant tumor uptake of whom: i) 8 patients were randomized in the Therapeutic part (3 patients in Arm A (370 MBq of ^90^Y) and 5 patients in Arm B (1110 MBq of ^90^Y)) and ii) 2 patients were not randomized and not treated with ^90^Y-OTSA-101 due to rapid general health status deterioration leading to early deaths (Fig. 1).

**Table 1:** Patients characteristics at baseline

			Imaging Part	Therapeutic Part	
			*N* = 20	*N* = 8	
			N (%)	Arm A	Arm B
				N	N
Number of Patients			20	3	5
Sex					
Men			10 (50.0%)	2	3
Women			10 (50.0%)	1	2
Age at inclusion (years)					
Mean			42.1	31.0	41.4
SD			13.68	10.44	13.59
Median			43.0	26.0	43.0
Range			21–67	24–43	21–57
PS (ECOG)					
0			8 (40.0%)	1	2
1			10 (50.0%)	2	2
2			2 (10.0%)	0	1
Primary tumor sites (at initial diagnosis)					
Upper limb			1 (5.0%)	0	1
Lower limb			8 (40.0%)	2	2
Trunck wall			5 (25.0%)	0	2
Internal trunck			4 (20.0%)	0	0
Head and neck			2 (10.0%)	1	0
Histological type					
Missing			1	0	1
Spindle cell			14 (73.7%)	3	2
Biphasic			2 (10.5%)	0	1
Poorly differentiated			3 (15.8%)	0	1
Histological grade at initial diagnosis	Grade 2		7 (35.0%)	3	2
	Grade 3		13 (65.0%)	0	3
	T	T1	5 (25.0%)	0	2
		T2	14 (70.0%)	3	3
		TX	1 (5.0%)	0	0
	N	N0	19 (95.0%)	3	5
		N1	1 (5.0%)	0	0
	M	M0	20 (100%)	3	5
Tumor depth					
Superficial			3 (15.0%)	1	2
Deep			17 (85.0%)	2	3
Disease status at inclusion					
Metastatic			18 (90.0%)	3	4
Locally advanced			1 (5.0%)	0	1
Both			1 (5.0%)	0	0
Surgery of the primary tumor					
Yes			18 (90%)	3	4
No			2 (10%)	0	1
Prior Radiotherapy					
Yes			15 (75.0%)	3	3
No			5 (25.0%)	0	2
Chemotherapy with Doxorubicin					
Yes, in monotherapy			5 (25.0%)	1	2
Yes, associated			15 (75.0%)	2	3
Chromosomal translocation site					
missing			1	0	0
SSX1			11 (57.9%)	1	4
SSX2			5 (26.3%)	1	0
Others			3 (15.8%)	1	1

Their clinical characteristics are described in Table 1. Briefly, there was an equal number of female and male, their median age was 43.0 years (min-max: 21–67). The most common histological subtype was spindle cell SS (14/20 patients (74%)) and SYT-SSX1 the most common molecular variant (11/20 (58%)). Almost all patients (19/20 patients) had metastatic disease at study entry, and lung was the most common site of metastasis. All patients had received prior chemotherapy with doxorubicin and the median number of previous regimen.

### Imaging studies, biodistribution and 2D dosimetry

All patients underwent at least 4 time points planar and SPECT-CT acquisitions. Planar and SPECT-CT images demonstrated physiological radiotracer accumulation predominantly in the liver, and at lower level in the blood pool, spleen, kidneys and intestines, and a very low bone marrow uptake. ^111^In-OTSA-101 lesions uptake was observed in all patients (at least Grade 1) with heterogeneous intensity on an inter-patient based analysis. Figure 2 shows examples of the highest radiotracer uptake in 3 patients on whole body planar acquisition (Fig. 2a) and on the correspondent SPECT-CT acquisition (Fig. 2b). Patients 3 and 8 demonstrated the most intense lesions uptake. Figure 3 shows the repeated plenary whole body scans for patient 8. Lung lesions uptake visually increased in time compare to mediastinal blood pool activity, consistent with specific tumor binding and internalization of the radiolabeled antibody.

**Fig. 2:** ^111^In-OTSA-101 visual uptake grading. Examples of ^111^In-OTSA-101 tumors uptake visualized in 3 patients on planar imaging (**a**) and assessed using visual scale applied on SPECT-CT acquisitions (**b**)

**Fig. 3:** ^111^In-OTSA-101 whole body planar scintigraphy repeated over time for patient 8 showing increasing lesions uptake compare to mediastinal blood pool

Tracer uptake became greater than mediastinum in at least one lesion for 9 patients (grade 3 or 4) as soon as 1 h after ^111^In-OTSA-101 injection for 2 patients and became obvious only at the last point acquisition for 3 patients. Some patients demonstrated large volume tumors with highly heterogeneous uptake consistent with tumor necrosis on CT (patients 12, 14 and 15). Tumor uptake was not correlated to tumor size and varied from one lesion to another in the same patient (Table 2). For example, patient 3 demonstrated a grade 2 in a 41 mm lesion in the right lung (Fig. 4a) as well as a grade 4 in a 40 mm left lung lesion (Fig. 4b).

**Table 2:** Minimal and maximal grade of ^111^In-OTSA-101 uptake in all the lesions for each patient. Only lesions greater than 1 cm were analyzed

Pt	Grade min	Grade max
pt 1	0	2
pt 2	0	2
pt 3	1	4
pt 4	1	1
pt 5	4	4
pt 6	0	2
pt 7	1	1
pt 8	2	4
pt 9	1	1
pt 10	1	3
pt 11	1	3
pt 12	4	4
pt 13	2	2
pt 14	3	3
pt 15	3	3
pt 16	1	1
pt 17	1	1
pt 18	1	1
pt 19	1	1
pt 20	2	4

**Fig. 4:** ^111^In-OTSA-101 SPECT-CT images performed at H72 in patient 3 showing a grade 2 lesion in the right lower lung lobe (**a**) and a grade 4 lesion in the left lower lung lobe (**b**)

Two-D dosimetry in the liver lead to a mean of 2.15 Gy [1.90–2.56 Gy] for the 3 patients in Arm A and 7.21 Gy [5.43–10.57 Gy] for the 5 patients in Arm B. Liver dose estimation was never to be greater than 20 Gy.

Overall, 10 patients were assessed as candidates to randomisation by the Steering committee including 9 patients with at least one lesion with tumor uptake ≥ Grade 3 and 1 patient with Grade 2 (Patient 2, first patient randomized).

### Safety

During the Imaging part, 19 of 20 patients (95%) experienced at least one adverse event (AE), 32 events were reported and 16 of 20 patients (80%) experienced at least 1 related AE. The most frequent related AEs (≥10%) were hypophosphatemia, lymphopenia, anemia, creatinine increased, hypomagnesemia, hemoptysis and leucopenia. The most frequent NCI CTCAE AE (≥10%) was lymphopenia. Of note only 1 patient experienced at least one related AE Grade ≥ 3: a Grade 3 lymphopenia. Thirteen SAEs were reported during the imaging part, all considered unrelated to study drug. No significant weight loss, deterioration of ECOG performance status, electrocardiogram changes were observed during the imaging part.

During the Therapeutic part, a total of 8 patients were randomized: 3 first patients received a single dose of 370 MBq of ^90^Y-OTSA-101, 4 patients received a single injection of 1110 MBq of ^90^Y-OTSA-101 and 1 patient received 2 injections of 1110 MBq of ^90^Y-OTSA-101 (Patient 01–003 who presented a SD at week12 was injected a second time at week 24). All patients experienced at least one AE in both study arms with a total of 90 related AEs (Table 3). Treatment-related AEs Grade ≥ 3 were seen in 4/5 patients in Arm B and 1/3 patients in Arm A. The most common related AEs were hematological toxicity (i.e. anemia, lymphopenia, thrombocytopenia, and neutropenia). Six SAEs were considered related to study drug during the therapeutic part, including one Suspected Unexpected Serious Adverse Reaction (SUSAR). Only one System Class Organ was represented: « Blood and lymphatic system disorders » with four cases of reversible lymphopenia and one case of thrombocytopenia. The reported SUSAR was a case of “Massive Hemoptysis leading to death” occurred in a 50 year-old female patient (Patient 3) 1.5 month after the 2nd injection of ^90^Y-OTSA-101 in a context thrombocytopenia (61,000 / mm3) and progressive lung metastases responsible of alveolar hemorrhage. The thrombocytopenia was probably related to the study drug, hemoptysis probably related to both study drug (as a complication of thrombocytopenia) and medical context of SS with progressive lung metastases.

**Table 3:** Treatment-related adverse events (AEs) observed during the therapeutic Part

	Arm A - 370 MBq		Arm B - 1110 MBq	
	*N* = 3		*N* = 5	
	Patients		Patients	
	N	%	N	%
All treatment-related AEs	3	(100.0%)	4	(80.0%)
Lymphopenia	3	(100.0%)	4	(80.0%)
Anemia	3	(100.0%)	3	(60.0%)
Leucopenia	1	(33.3%)	4	(80.0%)
Asthenia	2	(66.7%)	2	(40.0%)
Hemoptysis	1	(33.3%)	3	(60.0%)
Thrombopenia	1	(33.3%)	3	(60.0%)
Neutropenia	0	(0.0%)	3	(60.0%)
Anorexia	2	(66.7%)	0	(0.0%)
Creatinine increased	0	(0.0%)	2	(40.0%)
Hypokalemia	1	(33.3%)	1	(20.0%)
Nausea	1	(33.3%)	1	(20.0%)
Hypoalbuminemia	1	(33.3%)	0	(0.0%)
Hypophosphatemia	0	(0.0%)	1	(20.0%)
Hypoxemia	0	(0.0%)	1	(20.0%)
Vomiting	1	(33.3%)	0	(0.0%)
Weight loss	1	(33.3%)	0	(0.0%)
All treatment-related AE ≥ Grade 3	1	(33.3%)	4	(80.0%)
Lymphopenia	0	(0.0%)	3	(60.0%)
Thrombopenia	1	(33.3%)	2	(40.0%)
Anemia	1	(33.3%)	1	(20.0%)
Neutropenia	0	(0.0%)	2	(40.0%)
Asthenia	1	(33.3%)	0	(0.0%)
Hemoptysis	0	(0.0%)	1	(20.0%)
Hypoxemia	0	(0.0%)	1	(20.0%)
Leucopenia	0	(0.0%)	1	(20.0%)

### Tumor response

Tumor response was evaluated in the Therapeutic part (*n* = 8) at W6, W12 then every 12 weeks until EOS and assessed as per RECIST 1.1. No objective response was observed. The best overall response was SD in 3 patients (Table 4). Time to disease progression is summarised on Fig. 5. At Week 12, one patient (Patient 01–003) was assessed as SD in Arm B and received a 2nd injection of ^90^Y-OTSA-101 performed 6 months apart. This 49-year female patient remained progression-free for up to 21.4 weeks but died from haemoptysis related to lung disease progression.

**Table 4:** Best overall tumor response

Tumor Response as per RECIST v1.1	Arm A, *N* = 3	Arm B, *N* = 5
	Number of patients	Number of patients
CR	0	0
PR	0	0
SD	1	2
PD	2	3

*CR* complete response, *PR* partial response, *SD* stable disease, *PD* progressive disease as per RECIST 1.1

**Fig. 5:** Response to treatment assessed for each patient on time to disease progression in weeks after ^90^Y-OTSA-101 injection

### Pharmacokinetic & ADA

All patients, but one, had negative immunogenicity results (data not shown). The mean antibody serum half-lives were respectively 265.7 h (SD: 316.9; %CV: 119.3) in the first step, and 87.4 (SD: 66.6; %CV: 76.2) in Arm A and 61.8 (SD: 29; %CV: 46.9) in Arm B in the second step (S3) (Table 5). This led to a significantly reduced radiopharmaceutic exposure in the therapeutic part versus the imaging part.

**Table 5:** Phamacokinetics results for imaging part (A) and therapeutic part (B)

Parameter	Cmax	Tmax	T1/2	AUC C0-336^a^	CL	Vdss
Units	ng/mL	Hours	Hours	ng*Hours/mL	mL/Hours	mL
A. Imaging Part (*n* = 17)						
Mean	483.8	1.3	265.7	154,724	38.6	3311.9
S.D.	193.3	2.2	316.9	378,371	15.9	998.3
%CV	39.9	167.9	119.3	244.55	41.3	30.3
B. Therapeutic part (*n* = 8)						
ARM A (370 MBq, *n* = 3)						
Mean	365.4	0.00	87.4	42,106.7	255.4	4950.0
S.D.	240.3		66.6	38,489.5	391.9	4811.6
%CV	65.7		76.2	91.41	153.5	97.2
ARM B (1100 MBq, *n* = 4^b^)						
Mean	362.0	1.0	61.8	38,275.0	63.0	1787.7
S.D.	112.2	1.1	29.0	15,024.7	46.1	1040.5
%CV	31.0	115.5	46.9	39.25	73.1	58.2

NB: PK data were not analyzed for patients ID 01–0018, 01–019, 01–020 due to premature study and OTS-France closure

^a^or AUC extrapolated and BLQ concentration set to zero. ^b^data following the 2nd injection of patient 01–003 are included

## Discussion

We reported results of a FIH study with a radio-immuno-conjugate targeting *FZD10* in patients with advanced synovial sarcoma. The concept of vectorising cytotoxic and radionuclide has emerged 20 years ago when the first monoclonal antibodies as anti-cancer agents where approved, with some successes like radiolabelled anti-CD20 (Zevalin®) applied to non-Hodgkin-lymphoma as reviewed by Rizzieri [12] or more recently radiolabelled anti-PSMA applied to metastatic prostate cancer [13]. The overall aim of these anti-body drug conjugates (ADC) and radio-immunotherapy (RIT) is to use the specificity of monoclonal antibodies for their target to deliver a highly toxic payload (cytotoxic drug or radionuclide) to tumor cells, thus avoiding systemic toxicity of this payload. Key aspects in developing ADC/RIT are: 1) the target of the monoclonal antibody and its specificity, 2) payload and its individual cytotoxic potency, 3) the linker technology which will vary depending on the type of payload.

The linker technology was selected for maximum stability of the loaded antibody. In the present study we chose to have an assessment of target expression using FZD10-imaging with an ^111^In-labeled version of OTSA-101. Our study aimed to evaluate the in vivo ^111^In-OTSA-101 biodistribution and tumors biding rather than evaluating the maximal tolerated dose. As this was our main aim, we did not organize our study as a real 3 + 3 dose escalating study. Once biodistribution and tumors uptake would have been considered compatible with treatment, patients would be randomized to receive different doses of ^90^Y-OTSA-101, to give them more chance to receive an efficient dose. In standard dose escalation studies, as most responses occur between 80 and 120% of the Maximum Tolerated Dose (MTD), the first cohorts of patients are often treated with low sub-therapeutic dose and only few patients actually receive doses at or near the recommended therapeutic dose. Patients would rather beneficiate from a randomized study, giving more chance to patients to receive the effective dose treatment.

In the imaging part, we observed significant intra-patient and inter-patient differences in uptake intensity and uptake rates. Indeed, some patients had very low or no significant uptake of ^111^InOTSA-101 while in some patients we observed rapid uptake of target lesions. Although this heterogeneity was anticipated based on the preclinical data used as a basis for this study (8 of 13 SS patients had overexpression of *FZD10*, 4/13 had detectable expression and one patient had no detectable *FZD10* in the initial study by Nagayama et al. [3]), its importance was underestimated. The precise molecular or pharmacological mechanisms for these differences have not been explored in the current study. Another hurdle encountered during the preparation and conduct of this study, was the lack of validated immunohistochemistry (IHC) assay to assess *FZD10* expression on tumor cells. This lead us to propose the imaging part of the study as a biomarker, with the aim of reducing the number of patients exposed to Yttrium 90 to those most likely to benefit due to high in vivo expression. Due to the lack of available data at the time the study was initiated, we chose an arbitrary threshold of uptake based on a visual assessment of tumor uptake compared to background following Krenning’s grades applied for peptide receptors radionuclide therapy (PRRT) of endocrine tumors [14]. This visual scale allows for patients selection for PRRT as higher objective responses leading to longer survival and improved quality of life have been observed in case of higher grade tumors uptake [15]. Molecular imaging allows for a non-invasive whole body in vivo characterisation of the heterogeneity of tumors antigen or receptors expression between primary and metastases and as well as between metastases, supplementing the traditional role of using imaging for localizing and measuring disease. For example, it is currently used to conduct treatment of endocrine tumors as somatostatin receptors scintigraphy and ^18^F-FDG PET/CT are able to quantify sites of well and poorly differentiated disease, respectively, and therefore to treat more aggressively ^18^F-FDG PET/CT positive endocrine tumors [16]. Indeed, these whole body images are less influenced by biopsy bias. The in vivo expression of *FZD10* was not assessed on tumor biopsy as this procedure is exposed to sampling error and may not reflect the entire tumor cells heterogeneity. This is bypassed by whole body scintigraphies that allow tracking the radiotracer in the entire body and in every tumor. This is how we observed the difference of radiotracer uptake from one lesion to another and how we can proceed to dosimetry studies. Changes in radiotracers compounds can influence and change the biodistribution. This is the way we can improve the way they target tumors rather than normal tissues and thereafter, based on dosimetry studies, select the best molecule. This is the basis of theranostic in nuclear medicine [17, 18].

Kinetic of the lesions uptake reached maximum intensity as soon as 1 h post-injection in some patients while it would become obvious only on the latest acquisitions in others, consistent with specific tumor suptake. The tumors radiotracer retention observed confirmed radiotracer internalization. Some bulky tumors demonstrated heterogeneous tracer uptake as a result of the various tumors vascularizations, tumor necrosis depending on tumor size, the capacity of the antibody to diffuse into the tumors, the expression of FZD10, the antibody internalization. Thus, bystander effect or even the abscopal effect of radiopharmaceutical may occur only on a portion of the viable cells that would not show tracer uptake.

Tracer kinetic depends on tumors vascularization but also on tracer size. Antibodies are large molecules known to have poor tissues penetration and long circulating half-life. For this reason, more recent radionuclide therapy trials favour smaller radiolabelled vectors than antibody, such as fragments of antibodies (FAb), or mostly peptides, displaying more rapid tissue distribution and faster blood clearance, leading to almost no toxicity [19, 20]. Therefore, the development of FAb targeting *FZD10* may improve radiotracer kinetic and lesions uptake and reduce toxicity. It could be also possible to radiolabel it with a long physical half-life positron emitter such as Zirconium-89 (78.4 h) rather than Indium-111 to increase radiotracer detection in tumors by using Positron Emission Tomography (PET) camera, known for a better resolution than SPECT.

Overall loaded ^90^Y-OTSA-101 was well tolerated at all dose levels and no formal MTD was determined. No significant drug-related AE was observed with ^111^In-OTSA-101 but the injected doses were low in part 1 of the study to limit receptor occupancy by non-therapeutic antibody. In the second part of the study, the most common AEs were cytopenia and fatigue, with thrombocytopenia being the more problematic. Bone marrow suppression, which results in cytopenia, is most likely due to the exposure of the bone marrow to ^90^Y either bound to OTSA-101 during blood perfusion of bone marrow, or free ^90^Y which tends to accumulate in the bone marrow. Other isotopes such as Lutetium 177 (^177^Lu) for example are associated with reduced bone marrow suppression compared to ^90^Y [21, 22], due to a shorter mean pathway of less energetic electrons emitted (12 mm mean pathway in the water and Maximum 2270 Kev for 90Y vs 1.5 mm and 497 Kev for ^177^Lu).

We performed 2D dosimetry on ^111^In-OTSA-101 whole body acquisitions to estimate the absorbed dose of normal organs (liver, spleen, kidneys) when the patient would be treated with either 370 or 1110 MBq of ^90^Y-OTSA-101. As usually observed in RIT, liver was the most targeted normal organ by the radiolabeled antibody. However, the mean absorbed liver dose was calculated after Indium 111 in order to prevent reaching the 20 Gy Maximal Tolerated Dose (MTD) limit applied to external beam radiotherapy. When looking at liver toxicity, only one grade 1 bilirubin increase was reported in one patient treated by the lowest activity, contrasting with systematic bone marrow toxicity despite low visual bone marrow uptake and no diffuse medullary metastases in any patient. We recently reported the results of a 3D dosimetry based on Montecarlo simulations performed on these patients [23]. The calculated absorbed doses in the liver would range from 4.3 to 13 Gy, consistent with the 2D dosimetry results and the absence of liver toxicity. On the other hand, the absorbed dose in the bone marrow would be greater than 1.8 Gy for 5 patients, which is close to the MTD estimated around 2 Gy, partially explaining the observed bone marrow toxicity.

Efficacy of ^90^Y-OTSA-101 on tumors was mostly transient stabilized disease until disease progression. Most of the patients included in this phase I trial presented with bulky lung metastases. For this reason, a highly energetic electrons emitter such as ^90^Y would be more suitable to treat these lesions. However, these lesions were rapidly growing while radionuclide therapies demonstrate delayed response to treatment. This is well known for slowly progressive disease such as neuroendocrine tumors or thyroid cancers, with non-bulky disease. Moreover, the highly heterogeneous and mostly low ^111^In-OTSA-101 uptake observed in these tumors would lead to low absorbed doses in the tumors partially explaining the lack of treatment response especially in bulky tumors.

Altogether, when using ^177^Lu radiolabelled small molecules radionuclide therapy tend to be less toxic allowing increased injected doses in order to increase absorbed tumors doses. As a recent example, PSMA was first targeted with antibodies (J591) for diagnosis and therapeutic purpose of prostate adenocarcinoma. The maximum tolerated dose (MTD) due to marrow toxicity was 4 times lower when using ^90^Y-J591 than with ^177^Lu-J591 [22, 24]. For the past few years, high radiolabeled PSMA avid small molecules have been developed and used with great success for diagnosis and treatment. Different types of ^177^Lu-PSMA appeared to be highly tolerated with administered activities being twice the MTD of ^177^Lu-J591 with almost no grade 3–4 hematotoxicity in these populations of heavily pre-treated patients with bone metastases [19, 25, 26]. Moreover, dosimetry studies evaluate the absorbed tumors dose sometimes exceeding 100 Gy due to intense homogenous target lesions tracer uptake, which is far above the 10 Gy maximal absorbed dose in tumors we estimated on 3D [23].

## Conclusions

We confirmed the in vivo capacity of a new radiolabeled antigen targeting *FZD10* to get trapped in at least one metastasis in 20 patients presenting with metastatic synovial sarcoma. However, the ^111^In-OTSA-101 tumors uptake appeared highly heterogeneous and was considered intense enough to select patients for ^90^Y-OTSA-101 treatment in only half of the 20 patients included. A theranostic approach appeared feasible in a first in human phase I study in a very rare cancer using a national networking. Transient stable disease was observed in 5 of the 8 treated patients. However, as most of the patients presented significant hematotoxicity related to treatment, the use of small fragments of antibodies targeting *FZD10* radiolabeled with lower energetic electron emitter such as Lutetium 177 would be a favored option for further development.

## Abbreviations

ADC: anti-body drug conjugates
ADC: Anti-body Drug Conjugates
AE: Adverse Event
ANSM: Agence Nationale de Sécurité du Médicament
CLARA: Cancéropôle Lyon Auvergne-Rhône-Alpes
DLCO: Diffusing capacity or transfer factor of the Lung for Carbon monOxide
DTPA: Diethylene-Triamine-PentaAcetate
ECOG PS: Eastern Cooperative Oncology Group Performance Status
EDTA: EthyleneDiamineTetraAcetic acid
FACS: Fluorescence-activated cell sorting
FIH: First-In-Human
FVC: Force Vital Capacity
FZD10: Frizzled homologue 10
Gy: Grays
HACA: human anti-chimeric antibody.
HAMA: human anti-mouse antibody
IHC: immunohistochemistry
Kev: Kilo electro-volts
MAb: Monoclonal Antibody
MBq: Mega Becquerel
MTD: maximal tolerated dose
NCI-CTCAE: National Cancer Institute-Common Terminology Criteria
OTS: Onco Therapy Science
OTSA: OncoTherapy Science Antigen
PET: Positron Emission Tomography
PRRT: peptide receptors radionuclide therapy
PRRT: Peptide Receptors Radionuclide Therapy
PSMA: Prostate Specific Membrane Antigen
RECIST: Response Evaluation Criteria in Solid Tumours
RIT: radio-immunotherapy
RIT: Radio-ImmunoTherapy
SAE: Sever Adverse Event
SPECT: Single Photon Emission Computed Tomography / Computed Tomography
SS: Synovialosarcoma
SUSAR: Suspected Unexpected Serious Adverse Reaction
VEGF: Vascular endothelial growth factor
